# Efficacy of Butylphthalide in Combination with Edaravone in the Treatment of Acute Ischemic Stroke and the Effect on Serum Inflammatory Factors

**DOI:** 10.1155/2023/9969437

**Published:** 2023-04-11

**Authors:** Yan Li, Zhen Hong, Shaoquan Li, Songwang Xie, Junyong Wang, Jian Wang, Yongchang Liu

**Affiliations:** Department of Neurovascular Intervention, Cangzhou Central Hospital, Cangzhou, China

## Abstract

**Objective:**

To investigate the efficacy of butylphthalide combined with edaravone in the treatment of acute ischemic stroke and the effect on serum inflammatory factors.

**Methods:**

One hundred and sixty patients with acute ischemic stroke who attended the neurovascular intervention department of our hospital from May 2020 to June 2022 were enrolled as study subjects for prospective analysis and were equally divided into a control group and an experimental group using the random number table method, with 80 cases in each group. The control group was treated with edaravone injection, while the experimental group was treated with butylphthalide combined with edaravone. The disease was recorded to compare the efficacy, erythrocyte sedimentation rate, homocysteine, serum inflammatory factors including tumor necrosis factor-*α*, C-reactive protein and interleukin-6 levels, and the incidence of adverse reactions between the two groups.

**Results:**

The total effective rate of treatment in the experimental group was 90.0% (72/80), while that of the control group was 62.5% (50/80), the total effective rate of the experimental group was significantly higher than that of the control group, and the difference was statistically significant (*P* < 0.05). After treatment, the erythrocyte sedimentation rate, homocysteine level, and serum TNF-*α*, CRP, and IL-6 levels of patients in the experimental group improved compared with those before treatment, and the degree of improvement was better than that of the control group, and the difference was statistically significant (*P* < 0.05). After 3 months of treatment, a comparison of the incidence of adverse reactions in the two groups showed no statistically significant difference between the two groups (*P* > 0.05).

**Conclusion:**

The treatment of acute ischemic stroke with butylphthalide combined with edaravone has positive significance in improving blood circulation regulation and serum inflammatory factor levels and is reliable and worthy of clinical promotion.

## 1. Introduction

Ischemic stroke, also known as cerebral infarction, is a cerebrovascular disease caused by interruption of blood flow in the cerebral arteries and localised hypoxic-ischemic necrosis of brain tissue due to various causes [1]. Evidence has shown that ischemic stroke accounts for up to 70% of all strokes and is a common clinical cerebrovascular disease. This disease is characterized by high mortality, disability, and morbidity, and many patients suffer from various degrees of sequelae, which seriously impairs people's quality of life. Some findings show that the incidence of stroke is higher in the 50-60 age group than in other age groups, accounting for about 69.60% of strokes in China, and the number of patients with ischemic stroke has increased significantly with the increasing trend of aging in China. The occurrence of ischemic stroke, on the one hand, seriously affects the neurological function of patients [2], who are also prone to poststroke depression and cognitive dysfunction, and on the other hand, its high recurrence rate seriously threatens the physical and mental health of patients [3]. Therefore, it is important to pay more attention to ischemic stroke disease and to treat patients in a timely manner.

Pharmacological treatment is commonly prescribed, and the primary direction of clinical therapy is anti-inflammatory and anticoagulant, improving cerebral microcirculation [4]. Therapeutic drugs mainly contain blood pressure control, antiplatelet, anticoagulation, statins, etc. Although they can reduce the risk index and relieve patients' pain by improving the blood circulation in the ischemic area of the brain, protecting the damaged neurological function, and maintaining the normal operation of the body indicators, the effect of these drugs is not ideal. Butylphthalide, the third national innovative drug developed independently in China over a long period of time [5], which specifically targets several pathological aspects of acute ischemic stroke, improves perfusion in the ischemic region and helps to reestablish cerebral microcirculation and avoid brain mitochondrial damage; furthermore, it also has a significant role in promoting mitochondrial antioxidation and preventing thrombosis [6]. Edaravone is a widely used free radical scavenger in clinical practice, which can scavenge free radicals to inhibit the release of inflammatory factors, improve neurological function, and relieve the symptoms of acute ischemic stroke, but some patients may experience drug intolerance, triggering symptoms such as dizziness, headache, and nausea, resulting in unsatisfactory treatment outcomes.

Inflammatory doctrine mechanism is one of the important mechanisms in ischemic stroke. In the early ischemic phase of cerebral infarction, microglia are activated and their released inflammatory mediators, such as interleukin (IL) class and tumor necrosis factor-*α* (TNF-*α*), induce vascular endothelial cells to express adhesion molecules, etc., prompting circulating leukocytes (neutrophils, monocytes-macrophages, and lymphocytes) to roll and adhere to the injured vascular endothelium, migrate and cross the blood-brain barrier, and infiltrate and infiltrate the brain parenchyma. And through the release of a variety of proinflammatory mediators to further expand the local inflammatory response, it exacerbates the tissue damage at the site of injury and ischemic semidark zone, forming a state of rapid inflammation. Therefore, suppression of the inflammatory response is a key component in the treatment of ischemic stroke. The aim of this study was to investigate the efficacy of butylphthalide in combination with edaravone in the treatment of acute ischemic stroke and its effect on serum inflammatory factors, in order to provide a theoretical basis for clinicians to choose treatment measures.

## 2. Materials and Methods

### 2.1. Study Population

One hundred and sixty patients with acute ischemic stroke who attended the neurovascular intervention department of our hospital from May 2020 to June 2022 were enrolled and assigned 1 : 1 into either the control group or the experimental group using the random number table method. The control group was treated with edaravone injection, while the experimental group was treated with butylphthalide combined with edaravone.

The randomization was carried out using an online web-based randomization tool (freely available at http://www.randomizer.org/). For concealment of allocation, the randomization procedure and assignment were managed by an independent research assistant who was not involved in screening or evaluation of the participants. The original sample size calculation estimated that 50 patients in each group would be needed to detect a 3-point difference between groups in a 2-sided significance test with a power of 0.8 and an alpha error level of 0.05.

Informed consent was obtained from patients and signed prior to enrolment in the study. The study protocol was approved by the ethics committee of Cangzhou Central Hospital (Approval No. SKZ-X200325LS), and all processes complied with the *Declaration of Helsinki Ethical Guidelines* for clinical research.

### 2.2. Inclusion and Exclusion Criteria

#### 2.2.1. Inclusion Criteria

1. Patients who meet the relevant diagnostic criteria and brain imaging in the *Chinese Guidelines for the Treatment of Acute Ischemic Stroke* (2018)
2. Patients with a National Institutes of Health Stroke Scale (NIHSS) score of 4-18. The NIHSS score was used to assess neurological function before and after treatment in both groups, with a total score of 0 to 42, with higher scores resulting in poorer neurological function
3. Patients who have been treated in our neurology or emergency department for 2 weeks
4. Patients with complete relevant examination data before and after treatment

#### 2.2.2. Exclusion Criteria

1. Patients with intracranial haemorrhage (including substantial haemorrhage, subarachnoid haemorrhage, subdural/epidural haematoma, etc.)
2. Patients with a history of major head trauma or stroke within the past 3 months
3. Patients with active visceral haemorrhage
4. Patients with intracranial tumors and giant intracranial aneurysms
5. Patients on prothrombin inhibitors or factor Xa inhibitors within 48 hours and various sensitive laboratory abnormalities such as activated partial thromboplastin time (APTT), international normalized ratio (INR), platelet count, euglobulin lysis time (ECT), and prothrombin time (TT)
6. Patients with blood glucose < 2.8 mmol·L^−1^ or >22.22 mmol·L^−1^
7. Patients with imaging showing large infarcts (infarct area > 1/3 of the cerebral hemisphere)
8. Patients with severe combined cardiac, renal, or hepatic insufficiency

### 2.3. Treatment Methods

#### 2.3.1. Control Group

Patients in the control group were treated with edaravone (Shiyapharm Group Enbip Pharmaceutical Co., Ltd., H20100041, 100 mL) injection. 100 mg of 0.9% sodium chloride solution was mixed with 30 mg of edaravone injection, then administered intravenously to patients. Patients were injected twice daily for 2 weeks for a total of 1 course of treatment.

#### 2.3.2. Experimental Group

Patients in the experimental group were given butylphthalein (Centrum Pharmaceutical Co., H20050280) treatment based on the control group. 100 mg of 0.9% sodium chloride solution to 25 mg was mixed with butylphthalein injection, then administered intravenously to patients. Patients were injected twice daily for 2 weeks for a total of 1 course of treatment.

### 2.4. Efficacy Assessment Criteria

*Significantly effective*: after 14 days of treatment, clinical signs and symptoms completely disappeared or diplopia and aphasia signs improved significantly. In addition, patients showed significant improvement in neurological function and cerebral artery blood flow velocity, with a reduction in NIHSS score of >46%.

*Effective*: after 14 days of treatment, the patient showed some improvement in clinical symptoms, diplopia and aphasia, as well as improvement in neurological function and cerebral artery blood flow velocity, and an 18% to 45% decrease in NIHSS scores.

*Ineffective*: after 14 days of treatment, the patient's clinical signs and symptoms did not change significantly from baseline and did not meet the above criteria. In addition, the reduction in NIHSS scores was <18%.

The overall effective rate includes the rate of significantly effective and effective.

### 2.5. Outcomes

1. Blood rheological indexes. The erythrocyte sedimentation rate was measured by cone plate method, and homocysteine level was measured by coagulation method in both groups before and after interventions
2. Inflammatory factors. Serum tumor necrosis factor level was measured by ELISA-*α* method; moreover, interleukin-6 level and serum C-reactive protein level were measured by immunofluorescence method
3. Occurrence of adverse reactions. The incidence of postoperative adverse effects, including nausea and vomiting, dizziness and headache, elevated transaminases, and insomnia, was recorded and compared between the two groups. Incidence of adverse conditions = number of adverse events/total number of patients × 100%

### 2.6. Statistical Analysis

All data were of this study were collated and analyzed using SPSS 22.0. The mean difference between the two groups was tested using Student's *t*-test for normally distributed variables and Mann–Whitney *U* test for nonnormal variables. The measured data were expressed as mean ± standard deviation ($\bar{x}\pm s$) and compared using *t*-test. The count data was expressed as number of cases (%) and analyzed using the chi-square test. A value of *P* < 0.05 indicated that the comparison is statistically significant.

## 3. Results

### 3.1. Baseline Characteristics

In the experimental group, there were 43 males and 37 females, age 58.18 ± 8.25 years, onset time 20.47 ± 4.86 h. In the control group, there were 41 males and 39 females, age 58.53 ± 8.62 years, onset time 20.82 ± 4.61 h. In the control group, there were 41 males and 39 females, age 58.53 ± 8.62 years, onset time 20.82 ± 4.61 hours. The baseline characteristics were balanced between the two groups (*P* > 0.05).

### 3.2. Comparison of Clinical Efficacy

The total effective rate of treatment for patients in the experimental group (90.0% (72/80)) was significantly higher than that in the control group (62.5% (50/80)) (*P* < 0.05) (Table 1).

### 3.3. Comparison of Blood Rheological Indices

After 3 months of treatment, the erythrocyte sedimentation rate and homocysteine levels decreased in both groups, while the decrease in the experimental group was significantly greater than that in the control group (*P* < 0.05) (Table 2).

### 3.4. Comparison of the Levels of Inflammatory Factors

After 3 months of treatment, the serum levels of TNF-*α*, CRP, and IL-6 improved in both groups, and the improvement was greater in the experimental group than in the control group (*P* < 0.05) (Table 3).

### 3.5. Comparison of the Occurrence of Adverse Reactions

After 3 months of treatment, the incidence of adverse reactions between the two groups was similar (*P* > 0.05) (Table 4).

## 4. Discussion

Stroke seriously affects the quality of life of patients and places a heavy burden on society and families due to its high incidence, disability, recurrence, and poststroke depression [7]. The outcome of acute stroke determines the patient's prognosis, and poststroke depression is the most common mental health problem [8, 9]. The low rate of diagnosis and treatment of poststroke depression in China has seriously affected the recovery of stroke patients, thus increasing the recurrence rate and mortality of stroke. The etiology of acute ischemic stroke is complex, and its associated factors may include cerebral hemodynamic abnormalities, metabolic damage, and systemic factors [10].

Rapid restoration of blood supply to brain tissue, improvement of microvascular circulation and cerebral hypoxia and ischaemia, and repair of damaged nerve cells are currently the main tools and principles of clinical treatment [11]. Nerve cells in the “ischemic semidark zone” should be repaired as far as possible [12], because the lack of timely treatment and excitotoxic disturbances, secondary cell damage, inflammatory responses, and apoptosis in the “ischemic semidark zone” aggravate neurological deficit [13]. However, optimal treatment is often difficult to achieve through pathology alone [14], and therapeutic measures to prevent and control the progression of acute ischemic stroke have been unsuccessful in recent years [15], with many patients developing aphasia, paralysis, or dementia after treatment. Some scholars have found that atherosclerosis-induced stenosis is a common cause of thrombosis in posterior circulation ischemic stroke patients, slowing blood flow and putting blood in a hypercoagulable state, which in turn promotes thrombosis. In addition, emboli from other parts of the body are also very likely to be retained in the parts of the blood vessels with slow blood flow, thus causing secondary blockage. And when there is a large number of platelet aggregation, it will aggravate the narrowing of blood vessels and slow down the blood flow, resulting in a more serious state of blood hypercoagulation and eventually the formation of thrombus, leading to the lack of oxygen and ischemia in the brain. In clinical practice, a combination of different drugs is often required to prevent thrombotic progression and plaque dislodgement, aiming to open up collateral circulation, scavenge free radicals, reduce the production of inflammatory factors, rescue the ischemic semidark zone, reduce blood viscosity, dilate blood vessels, and enhance cerebral perfusion as well as reduce the extent of brain tissue damage in the shortest possible time [16], which are the focus of comprehensive treatment. It has been found that the use of copper blue protein hydrolysate alone in the treatment of ischemic cerebrovascular disease was not satisfactory, with poor improvement in patients' blood rheological parameters, and more effective treatment options need to be sought [17].

Butylphthalide is a new drug derived from celery seed, which is a synthetic racemic n-butylphthalide that reduces brain cell death, protecting mitochondrial function and improving perfusion in ischemic areas [18]. Butylphthalide treatment for acute cerebral infarction promotes improvement in neurological deficits and improves impairment of central nervous function. Related studies have demonstrated that butylphthalide improves lipid metabolism and blood rheology, inhibits spasm, promotes cerebral blood circulation, and helps to improve hypoxic-ischemic nerve cell function. In furtherance, d_1_-3-n-butylphenyl peptide in butylphthalide improves brain microcirculation, enhances brain cell activity, and is effective against cerebral ischemic diseases [19, 20]. Edaravone is a cerebroprotective agent that reduces symptoms of cerebral ischaemia and oedema and penetrates the blood-brain barrier rapidly to reach the tissues [21], effectively reducing local cerebral blood flow around the infarct site and improving neurological function in patients with acute cerebral infarction.

The results of this study revealed that the overall efficiency of the experimental group was significantly higher than that of the control group, and the improvement of blood rheological indexes in the experimental group was greater than that in the control group after treatment, and the difference was statistically significant, which proved that butylphthalide combined with edaravone could help regulate blood circulation and improve the efficacy of treatment. Atherosclerosis is the main pathological basis for the development of stroke, which leads to thickening and hardening of the arterial wall, causing luminal narrowing and occlusion, which in turn slows blood flow, increases thrombosis, leads to vascular obstruction, impairs endothelial function, and leads to persistent progression of the disease [22]. In this analysis, combined application of butylphthalide treatment can promote stroke disease control and protect neurological function by inhibiting atherosclerosis, improving carotid blood flow status, and regulating vascular endothelial function. Its mechanism of action mainly lies in the fact that butylphthalide can selectively inhibit arachidonic acid activity, anticoagulate, and antithrombin generation and stabilize cerebral blood flow, while scavenging oxygen free radicals, inhibiting neuronal apoptosis, increasing antioxidant enzyme activity, and promoting damaged blood vessel repair, thereby effectively restoring cerebral blood flow and neurological function [23]. Edaravone is conducive to protecting brain nerve cells, inhibiting lipoprotein oxidation, and scavenging free radicals.

TNF-*α* is an important effector molecule in the inflammatory cascade, plays an important role in the inflammatory response of the central nervous system, is involved in the process of arterial vascular disease, and increases the risk of stroke if levels are too high [24]. CRP is a nonspecific inflammatory marker reflecting chronic inflammation in the body; under normal conditions, CRP levels are relatively extremely low, while its abnormally high expression leads to monocyte chemotaxis and promotes atherosclerosis, resulting in vascular disease. IL-6 is an inflammatory mediator that mediates astrocyte expression and promotes protein precursor protein synthesis, which could trigger overgrowth of dystrophic axons in the brain, leading to the formation of neuroinflammatory plaques that lead to cognitive dysfunction [25]. The results of this study indicated that serum TNF-*α*, CRP, and IL-6 levels in the experimental group improved more after treatment, and the difference was statistically significant. The above experimental results show that butylphthalide combined with edaravone could help regulate serum inflammatory factors and reduce inflammation in stroke patients and possess a certain degree of safety.

Hcy is a reactive amino acid synthesised during methionine metabolism that induces platelet adhesion to endothelial cells and enhances coagulation [26]. It has been reported that higher Hcy levels are associated with a poorer survival prognosis in Caucasian and Asian patients with acute ischemic stroke, and on this basis, Hcy may be an independent predictor of a poorer survival prognosis after acute ischemic stroke. The results of this study indicated that the combination of butylphthalide and edaravone provided additional benefits to patients with acute ischemic stroke, improving neurological damage and reducing plasma Hcy levels more effectively.

Despite the fact that there are also a number of studies on stroke, this study was distinguished from conventional clinical studies by evaluating not only the changes of butalbital combined with edaravone on patients' symptoms and seriousness from a subjective point of view. It also observed the efficacy of butalbital combined with edaravone on inflammatory factors and blood coagulation based on the current hot neuroimmunological indicators to provide clinicians with a deeper understanding of the impact of this treatment modality.

However, there are still some limitations in this study. The cases were obtained from the inpatients of neurovascular intervention department of our hospital, which is a single-center study with a small sample size, and the observation period is not long enough, so the clinical results might be biased. This study did not consider the influence of the patients' physical constitution on the drug dose and absorption, so there is no adjustment of the use of butalbital and edaravone, and the possible confounding factors cannot be excluded. In addition, this study is a clinical study, and there is a lack of animal experiment, lacking more scientific basis. In future studies, ongoing studies are required to further expand the source of cases and sample size, as well as involve more related indicators, such as safety, and extend the observation period and follow-up, to secure more reliable data.

## 5. Conclusion

In summary, the combination of butylphthalide and edaravone in the treatment of acute ischemic stroke has a positive effect on the regulation of blood circulation and serum inflammatory factor levels in patients and is safe and worthy of clinical promotion.

## Figures and Tables

**Table 1:** Comparison of clinical outcomes between the two groups of patients.

Group	Cases	Markedly effective	Effective	Ineffective	Total effectiveness
Experimental group	80	40	32	8	72 (90.0%)
Control group	80	18	32	30	50 (62.5%)
*x* ^2^	—				16.704
*P*	—				≤0.1

**Table 2:** Comparison of blood rheological parameters between the two groups.

Group		Erythrocyte sedimentation rate (mm/h)	Hcy (*μ*mol/L)
Experimental group (*n* = 80)	Before treatment	25.76 ± 3.52^#^	19.32 ± 6.09^#^
	After treatment	11.86 ± 1.25^∗^	12.76 ± 3.42^∗^
Control group (*n* = 80)	Before treatment	26.13 ± 3.74^#^	20.09 ± 7.26^#^
	After treatment	20.61 ± 2.87^∗^	16.74 ± 4.63^∗^

Notes: # represents *P* > 0.05; ^∗^ represents *P* < 0.05.

**Table 3:** Comparison of inflammatory factor levels.

Group		Tumor necrosis factor-*α* (*ρ*g/mL)	C-reactive protein (mg/L)	Interleukin-6 (*ρ*g/mL)
Experimental group (*n* = 80)	Before treatment	30.51 ± 1.53^#^	1.89 ± 0.23^#^	123.86 ± 12.85^#^
	After treatment	18.43 ± 1.26^∗^	0.77 ± 0.19^∗^	49.93 ± 4.82^∗^
Control group (*n* = 80)	Before treatment	30.23 ± 1.27^#^	1.89 ± 0.21^#^	124.82 ± 11.53^#^
	After treatment	21.74 ± 1.33^∗^	1.21 ± 0.23^∗^	78.52 ± 7.09^∗^

Notes: # represents *P* > 0.05; ^∗^ represents *P* < 0.05.

**Table 4:** Comparison of the incidence of adverse reactions between the two groups.

Group	*n*	Nausea and vomiting	Dizziness and headache	Elevated transaminases	Insomnia	Total incidence
Experimental group	80	2	1	1	2	6 (7.5%)
Control group	80	1	1	3	2	7 (8.7%)
*χ* ^2^						0.084
*P*						0.772

## Data Availability

All data generated or analyzed during this study are included in this published article.
